This article has been retracted.

# Study on the Mechanism of Xiaotan Sanjie Recipe in the Treatment of Colon Cancer Based on Network Pharmacology

**DOI:** 10.1155/2022/9498109

**Published:** 2022-08-05

**Authors:** Xiao-wei Wang, Ci-an Zhang, Min Ye

**Affiliations:** Department of Traditional Chinese Medicine, Changzheng Hospital, Second Military Medical University, Shanghai 200003, China

## Abstract

The aim of the study is to investigate the mechanism of action of Disulfiram against colon cancer through a network pharmacology approach. The targets were then imported into the Cytoscape 3.7.2 software to construct a network of active ingredient targets and were imported into the STRING database to construct a protein-protein interaction (PPI) network, and the Bisogenet plug-in in Cytoscape 3.7.2 was used for network topology analysis. Gene ontology (GO) enrichment analysis and Kyoto Encyclopedia of Genes and Genomes (KEGG) enrichment analysis were performed on the potential targets of Yiqi and Baiyu Tang for colon cancer using the R-language Bioconductor platform, and the results were imported into Cytoscape 3.7.2 to obtain KEGG network relationship maps. Molecular docking software Autodock Vina was used to map the core targets to the active ingredients. A total of 119 chemical components and 694 disease targets were obtained, including 113 intersecting targets. The key targets included AKT1 and TP53, and GO functional analysis mainly related to ubiquitination and apoptosis, etc. KEGG analysis showed that the treatment of colon cancer with Ganchenzan mainly acted through cancer-related signaling pathways such as AGE-RAGE and P13K-Akt, and the molecular docking results showed the best binding performance with TP53.

## 1. Introduction

Colon cancer is the fourth leading cause of cancer-related deaths in the world. In symptomatic patients, 60%–70% of confirmed cases are found in the late stage of the disease [1]. At present, the treatment of colon cancer is a comprehensive treatment method led by surgery and supplemented by chemotherapy and radiotherapy [2].

However, the antitumor drugs in chemotherapy inhibit and kill not only tumor cells but also normal cells [3]. Therefore, efficient and low toxicity antitumor drugs are urgently needed. Medicine Food Homology Species demonstrate critical, low toxicity antitumor properties with prospective applications in tumor treatment. The study is aimed at providing theoretical support for the development and utilization of these low toxicity, plant-based drugs.

Network pharmacology is one of the achievements of big data research. Different from traditional single component and single target thinking, its multicomponent, multitarget, and multichannel network building thinking is more suitable for the complex characteristics of traditional Chinese medicine compound. Networked pharmacology, as a new method, provides a lot of information about compounds, targets, diseases, etc., for pharmacological research of unique Chinese drugs and compounds. It can analyze the mechanism of action of traditional Chinese drugs from the perspective of modern pharmacology and also provide help for the research and development of new Chinese drugs and new dosage forms. At the same time, the network pharmacological method can be used to demonstrate the general concept, differentiation and treatment of the syndrome, different treatments for the same disease, and the same treatment for different diseases in the theory of traditional Chinese medicine, so as to provide data support for accurate medical treatment of traditional Chinese medicine. It can also demonstrate the compatibility theory of monarch, minister, assistant, drug pair, mutual requirement, mutual assistance, mutual assistance, etc., and clarify the role and changes of drug toxicity in prescription due to compatibility.

Xiaotan Sanjie Recipe (*Pinellia ternata*, Nan-xing, Tianlong, *Scorpio*, tangerine peel, *Galli Gigerri Endothelium Corneum*, and Zhi Gan Cao) has been Professor Wei Pinkang's empirical prescription for treating gastrointestinal (GI) tumors for more than 40 years. Preliminary clinical studies show that Xiaotan Sanjie Recipe can effectively improve the card score in patients with advanced GI tumors and prolong the survival time [4]. Some studies have found that Xiaotan Sanjie Recipe can inhibit the proliferation of human colorectal cancer HCT116 cells by promoting cell apoptosis in the tumor cells [5]. Xiaotan Sanjie Recipe was found to inhibit the proliferation of colon cancer stem cells, block the cell cycle and induce apoptosis *in vitro*, and inhibit the growth of colon cancer stem cells that are transplanted as tumors *in vivo*. Tumor-bearing mice subjected to high doses of the recipe showed prolonged survival time and improved survival rate. *In vivo* and *in vitro* settings show that the recipe can significantly inhibit the Wnt/*β*-catenin pathway and downregulate the transcription of target genes and, thereby, the expression of some colon cancer stem cell markers. The upstream regulation mechanism leading to inhibition of pathway activity may follow either of the two mechanisms: The first is caused by inhibition of AKT activity, activation of GSK-3*β* function, and degradation of *β*-catenin; the second mechanism likely involves widely downregulating the expression of receptors and ligands that upregulate the Wnt/*β*-catenin pathway, thereby reducing pathway receptor-ligand response [6, 7]. Although the active components of Xiaotan Sanjie Recipe have been extensively studied, there are few studies on the traditional Chinese medicine (TCM) compound Danshen Decoction.

## 2. Materials and Methods

### 2.1. Screening of Target Components of Xiaotan Sanjie Recipe

TCMSP and TCMID, the pharmacological platforms of the TCM system, enabled finding the active chemical components of the Xiaotan Sanjie Recipe (*Pinellia ternata*, Nan-xing, Tianlong, *Scorpio*, tangerine peel, *Gigerri Endothelium Corneum*, and Zhi Gan Cao). TCMSP is set with oral bioavailability (OB) ≥ 30% and druglikeness (DL) ≥ 0.18 for screening [5]; TCMID is screened in Swiss adme. Per the screening conditions, GI absorption during pharmacological treatment was high, and more than two parameters in druglikeness were rated as “yes.” The ineffective components were removed, and the active components of TCM in the Xiaotan Sanjie Recipe are obtained. Potential protein targets are obtained through the Swiss target prediction database, and the screening condition was set at probability ≥ 0.1. The screened protein targets, like the protein game, were converted into standardized gene names in the UniProt database.

### 2.2. Screening of Colon Cancer-Related Targets

OMIM and GeneCards databases were searched to identify the target genes related to colon cancer using the keyword “colon cancer.” Multiple target genes were retrieved from the GeneCards database. Targets were filtered per the score value: the higher the score, the stronger the correlation between the target and the disease.

### 2.3. Acquisition of Effective Targets and Drawing of the Venn Diagram

A Venn diagram was drawn to determine the intersection of the Xiaotan Sanjie Recipe targets and colon cancer targets. The targets in the intersection were identified as effective targets of Xiaotan Sanjie Recipe in colon cancer treatment.

### 2.4. Construction and Analysis of Active Component-Effective Target Network

The active ingredients from the Xiaotan Sanjie Recipe and the identified effective target genes were introduced into the Cytoscape 3.7.2 [6] software and the drug active component-effective target network diagram was obtained.

### 2.5. Construction of Protein Network

The effective targets of the Xiaotan Sanjie Recipe and colon cancer were imported into the STRING database to construct a protein interaction network. Data with reliability ≥ 0.900 were imported into the Cytoscape 3.7.2 software in tsv format for visual analysis, and protein-protein interaction (PPI) data were extracted using R programming. Connection points of core genes were identified, and a histogram of the first 30 core genes was drawn.

### 2.6. Enrichment Analysis of Target Function and Pathway

The R software (https://www.r-project.org/) and its background object database https://org.hs.eg/.db were assessed to obtain the gene ID (entrezID) of potential action targets, and then, the program packages of DOSE, clusterProfiler, and path view accessed using the Bioconductor open-source software were used to conduct gene ontology (GO) function enrichment analysis on the identified potential active targets, which included the following three functions: biological process (BP), cellular component (CC), and molecular function (MF). *P* value and *q* value cutoffs were set at 0.05. Each category was sorted according to its significance, and the top 10 enrichment items were displayed in the form of a histogram and bubble chart.

### 2.7. Docking of the Main Active Ingredients and Target Molecules of Xiaotan Sanjie Recipe

The targets of Xiaotan Sanjie Recipe on colon cancer were searched the PDB database saved in the pdb format. The ligands were stored in mol2 format with the top 2 compounds after topological analysis (degree value). The potential targets Xiaotan Sanjie Recipe colon cancer were connected with the main compounds in Xiaotan Sanjie Recipe by AutoDockTools-1.5.6.

## 3. Results

### 3.1. Acquisition of Active Components and Related Targets of Xiaotan Sanjie Recipe

Taking screening conditions as OB ≥ 30% and DL ≥ 0.18, GI absorption≥two yes in DL, and 119 active components in the phlegm powder were eliminated. 1001 TCM targets were retrieved by TCMSP and TCMID (see Table S1 for active components).

### 3.2. Acquisition of Colon Cancer-Related Targets

The disease-related genes were obtained from GeneCards and OMIM databases. Targets with a score greater than the median were considered potential targets for disease treatment. Combined with the relevant targets retrieved from the OMIM database, the duplicate values were deleted after merging, and finally, 694 colon cancer-related targets were obtained.

### 3.3. Venn Drawing

Using the Venn tool in TBtools, the intersection of Xiaotan Sanjie Recipe target and colon cancer target was obtained, and 133 intersection targets were obtained. The results are shown in Figure 1.

### 3.4. Construction of an Active Component-Effective Target Network Diagram of Xiaotan Sanjie Recipe

Cytoscape 3.7.2 was used to construct the active component and effective target network of Xiaotan Sanjie Recipe, as shown in Figure 2. The network topology parameters of Xiaotan Sanjie Recipe in the treatment of colon cancer were calculated by the software to evaluate the importance of the active components and effective targets. The results showed that quercetin, gingerol, nicotinic acid, and other active components of the recipe can act on multiple targets. These components may be the main active components of Xiaotan Sanjie Recipe in the treatment of colon cancer.

### 3.5. Construction of Protein Network

Use Venn tool in TBtools to intersect the target between Xiaotan Sanjie Recipe targets and colon cancer, as shown in Figure 1. Upload the intersection target to STRING database, set the confidence level ≥ 0.9, and obtain the PPI network diagram of the target. Import the data into Cytoscape 3.7.2 to draw the protein network diagram. The bigger the node, the greater the corresponding degree value. According to the degree value, judge the location in the network. According to Figure 3, the targets in the center of the network are TP53, AKT1, Myc, etc.

### 3.6. Enrichment Analysis Results of Target Function and Pathway

Using the R software, GO annotation of effective targets was analyzed to select the top 20 results among BP, CC, and MF, respectively. BP enriched by these targets was mainly related to cellular oxidative stress, apoptosis signal, reproductive structure development, steroid hormones, and so on. MF mainly involved ubiquitinated protein ligase binding, cytokine corresponding binding, transcription factor complex, etc. CC mainly involved nuclear chromatin, membrane raft, and micromembrane area. These results are shown in Figure 4(a). KEGG database enabled to enrichment and analysis of 174 signal pathways, including the AGE-RAGE signaling pathway, TNF signaling pathway, P13K-AKT, and IL-17. The first 20 pathways were selected for visualization. These results are shown in Figure 4(b).

### 3.7. Molecular Docking Results of Active Components of Xiaotan Sanjie Recipe

After topological analysis and calculation, the main compounds of the Xiaotan Sanjie Recipe were obtained. The potential targets and main compounds of Xiaotan Sanjie Recipe acting on colon cancer were docked using AutoDockTools-1.5.6. Greater stability in the conformation of the ligand and receptor binding was predicted to have a greater probability of drug action. Per the degree value, the top two key targets were found to be serine/threonine kinase (AKT1) and TP53 tumor protein (TP53). Using AutoDock Vina for molecular docking of the components, the following results were observed between ligand small molecules and receptor proteins: binding energy < −4.25 kcal/mol suggested a certain binding activity; binding energy < −5.0 kcal/mol shows good binding activity; binding energy < −7.0 kcal/mol indicates strong binding activity [8]. The binding energies of quercetin and gingerol to the core target were found to be -7.7 and -4.6 kcal/mol, respectively, indicating that the drug recipe has a strong binding activity to the target. The specific docking results are shown in Figure 5.

## 4. Discussion

The number of colon cancer has seen a sharp increase, especially in younger patients, possibly owing to eating habits and lifestyle [9]. About 1 million new cases of colon cancer are annually reported worldwide, and the mortality rate is as high as 40% [10]. Currently, colon cancer treatment involves comprehensive care and is based on surgery. Developing new, targeted drugs for colon cancer treatment is, therefore, warranted.

Herbal TCMs have shown good tumor curative properties. Active components from Herbal TCMs have been screened for preventing and treating colon cancer and have shown encouraging scientific significance and application prospects [11]. The pathogenesis of colon cancer is not caused by a single target, but rather by multiple targets working cohesively and these targets keep changing based on the different stages of disease development; this mechanism is aligned with the characteristics and connotation of TCM, i.e., multitarget, multicomponent, and multiregulative [12, 13]. Currently, data mining, network pharmacology, and computer-aided drug design are playing an important role in the modernization of TCM remedies.

In this study, the main active components of Xiaotan Sanjie Recipe in colon cancer treatment were found to be quercetin, kaempferol, and luteolin. Quercetin is a natural small molecule flavonoid. Relevant pharmacological studies have shown that quercetin plays an anticolon cancer role by inducing apoptosis in HCT116 colon cancer cells by regulating the Sestrin 2-AMPK-mTOR signal pathway [14]. Kaempferol inhibits the proliferation of human colon cancer SW480 cells by inducing cell cycle arrest and p53-mediated mitochondrial apoptosis pathway [15]. Luteolin has been shown to inhibit colon cancer metastases by inhibiting the proliferation, migration, and epithelial-mesenchymal transformation of colon cancer cell HT-29 [16].

The core proteins determined by PPI were TP53, AKT1, Myc, EGFR, CCND1, JUN, CASP3, STAT3, etc. Among these, AKT1 and AKT2 gene knockout have been shown to reduce metastasis and growth of colon cancer [17].

The KEGG pathway enrichment analysis results showed that the main signal pathways in the treatment of colon cancer using Xiaotan Sanjie Recipe included the cancer pathway, the PI3K-AKT signal pathway, and the apoptotic pathway. PI3K-AKT signaling pathway plays an important role in tumor growth and progression [18, 19]. The overactivation of the PI3K/AKT signaling pathway leads to the decreased expression of tumor suppressor protein p53, leading to increased protein synthesis and tumor cell proliferation and therefore inhibition of cell apoptosis [20]. Tang Jian et al. [21] found that the proliferation of human colon cancer HT-29 cells can be inhibited by inhibiting the PI3K/AKT signaling pathway; this is achieved by inhibiting the downstream expression of the P-glycoprotein transduction pathway and blocking the cell cycle in the G1 phase. Currently, there is limited literature reporting the mechanism of Xiaotan Sanjie Recipe in the treatment of colon cancer. Some studies have revealed that its mechanism may be related to cell apoptosis. Xiaotan Sanjie decoction inhibits interleukin-8-induced metastatic potency in gastric cancer, blocks the cell cycle, and induces apoptosis *in vitro* [22]. However, other pathways and possible mechanisms of antitumor activity need further analysis and experimental verification.

Of course, network pharmacology has many limitations [23]. This is not a simple supplement to the chemical components of traditional Chinese medicine [24]. The content and concentration of traditional Chinese medicine affect the therapeutic effect. The establishment of any theoretical model does not depend on experimental verification, nor does it depend on the laboratory verification of pharmacological research of traditional Chinese medicine network. Ye et al.'s research discusses progress and perspectives in network pharmacology, focusing on the discovery of out-of-target drugs, the identification of disease-associated proteins, and the analysis of the pathway to clarify the relationships between drug targets and disease-associated proteins [25]. Vogt and Mestres's research introduces two approaches to measure the loss of information associated with bipartite network projection. The application to two structurally distinct cases in network pharmacology, namely, bipartite networks target drug and disease gene, confirms that the main determinant of information loss is the degree of vertices omitted during single-party projection [26]. Li et al.'s research highlighted the necessity and proposed the strategies for improving the methodology of conventional network pharmacology [27]. The accuracy and reliability of prediction can only be verified by combining network-based prediction with experimental verification and biological experiment with network pharmacological prediction. Of course, this does not depend on the cooperation and communication between online pharmacology groups.

## 5. Conclusion

In conclusion, using the network pharmacology method, this study preliminarily attempts to predict the possible mechanism of Xiaotan Sanjie Recipe in treating colon cancer. The study also reveals that Xiaotan Sanjie Recipe treats colon cancer from multicomponent, multitarget, and multichannel mechanisms and provides a basis for further experimental verification and clinical research. There are still some limitations in this study, such as different databases with different targets, which may be missing.

## Figures and Tables

**Figure 1:** Venn diagram of intersection target of Xiaotan Sanjie Recipe and colon cancer.

**Figure 2:** Active component-effective target network diagram of Xiaotan Sanjie Recipe.

**Figure 3:** Target intersection and PPI network diagram: (a) PPI network diagram; (b) core gene map; (c) protein interaction diagram.

**Figure 4:** Enrichment analysis of Xiaotan Sanjie Recipe in the treatment of colon cancer: (a) GO enrichment analysis; (b) KEGG enrichment analysis.

**Figure 5:** Molecular docking mode diagram: (a) docking diagram of quercetin and TP53; (b) docking diagram of gingerol and AKT1.

## Data Availability

The datasets used and analyzed during the current study are available from the corresponding author on reasonable request.

## Supplementary Materials

Supplementary Materials In TCMSP and TCMID databases, 119 active components in the phlegm powder were eliminated and were obtained using OB ≥ 30% and DL ≥ 0.18; the active components are shown in the Supporting File (Table S1, supporting information). A total of 1001 TCM targets were listed as Table S1 for active components.
